The article "High Antipredatory Efficiency of Insular Lizards: A Warning Signal of Excessive Specimen Collection?" was published in 2011. Journal: PLoS One.

# High Antipredatory Efficiency of Insular Lizards: A Warning Signal of Excessive Specimen Collection?

**DOI:** 10.1371/journal.pone.0029312

**Published:** 2011-12-28

**Authors:** Miguel Delibes, María del Carmen Blázquez, Laura Soriano, Eloy Revilla, José Antonio Godoy

**Affiliations:** 1 Department of Conservation Biology, Estación Biológica de Doñana, Consejo Superior de Investigaciones Científicas, Sevilla, Spain; 2 Department of Environmental Planning and Conservation, Centro de Investigaciones Biológicas del Noroeste, La Paz, Baja California Sur, México; 3 Department of Integrative Ecology, Estación Biológica de Doñana, Consejo Superior de Investigaciones Científicas, Sevilla, Spain; University of Jyväskylä, Finland

## Abstract

We live-captured lizards on islands in the Gulf of California and the Baja California peninsula mainland, and compared their ability to escape predation. Contrary to expectations, endemic lizard species from uninhabited islands fled from humans earlier and more efficiently than those from peninsular mainland areas. In fact, 58.2% (n = 146) of the lizards we tried to capture on the various islands escaped successfully, while this percentage was only 14.4% (n = 160) on the peninsular mainland. Separate evidence (e.g., proportion of regenerated tails, low human population at the collection areas, etc.) challenges several potential explanations for the higher antipredatory efficiency of insular lizards (e.g., more predation pressure on islands, habituation to humans on the peninsula, etc.). Instead, we suggest that the ability of insular lizards to avoid predators may be related to harvesting by humans, perhaps due to the value of endemic species as rare taxonomic entities. If this hypothesis is correct, predation-related behavioral changes in rare species could provide early warning signals of their over-exploitation, thus encouraging the adoption of conservation measures.

## Introduction

Rare species are particularly interesting to hunters, pet owners, curators of museum or natural history collections and scientists. As a consequence, rarity-fuelled demand may reduce population numbers, making these species even rarer and more desirable, thus driving them towards extinction [1], [2]. This fact may explain, at least partially, the disappearance of many species shortly after their discovery [3]. Therefore, it is important to recognize early signals of excessive exploitation, as they could encourage the adoption of cautionary measures. We believe that animal behavior is a particularly useful indicator of human disturbance [4]. In this study, we describe and discuss a behavioral change in a group of endemic lizards that could be interpreted as a response to collection pressure.

The so-called “evolutionary ecology of fear” [5] has received a great deal of attention over the last few years. At the intraspecific level, it is generally accepted that the behavior of individuals along a “shy-bold continuum” is predictable and can be related to the current and historical intensity of predation, as well as to other factors (e.g., habitat, availability of refuges, type of predator, etc.) [6]. For instance, in the case of lizard species it has been demonstrated that the introduction of domestic cats increases the wariness of previously naïve *Tropidurus* spp. in the Galapagos Islands [7]. Similarly, antipredatory behavior (flight initiation distance, distance fled and hiding time) varies dramatically in *Podarcis lilfordi* and *Ctenosaura hemilopha* individuals living with and without predators [8], [9] and *Aspidoscelis tesselata* adaptively changes fleeing speed and wariness in more risky habitats [10]. Thus, it should be possible to interpret any noticeable spatial or temporal change in the antipredator behavior of a particular group of lizards in terms of the predation pressure and the surrounding conditions [11].

In the present study we explore the link between antipredator behavior and predation pressure using the Orange-throated whiptail (*Aspidoscelis hyperythra* group) as a model species. This group occupies several islands in the Gulf of California and most of the Baja California peninsula mainland. The Gulf of California is an amazing laboratory of biogeography and evolution [12], where many species have been well-studied from a phylogenetic and taxonomic point of view. One of these species is the Orange-throated whiptail, a small lizard ∼6 g in weight (individuals are larger on Cerralvo Island). As many as seven closely related species are recognized in the group [13], with a distinct species found on the peninsular mainland and one on each of six different islands (Table 1).

**Table 1:** Capture results and characteristics of sampling localities.

Locality reference	Insular endemic (1)/No endemic (0)	Cats (1)/no cats(0)	Number of lizards captured (regenerated tails)	Number of lizards chased but not captured	*Aspidoscelis* species (*sensu* Grismer,1999)
Islands					
Coronados	0	0	8 (5)	7	*A. hyperythra*
Carmen	1	1	7 (4)	12	*A.carmenensis*
Montserrat	1	0	2 (0)	17	*A. picta*
San José	1	1	13 (4)	1	*A. danheimae*
San Francisco	1	0	7 (2)	9	*A. franciscensis*
Espíritu Santo	1	1	12 (8)	16	*A. espiritensis*
Cerralvo1	1	1	6 (5)	9	*A. ceralbensis*
Cerralvo 2	1	1	6 (1)	14	*A. ceralbensis*
Mainland					
Pur	0	1	3 (2)	0	*A. hyperythra*
Rde	0	1	5 (3)	0	*A. hyperythra*
Agv	0	1	5 (1)	2	*A. hyperythra*
Ins	0	1	3 (1)	0	*A. hyperythra*
Ihu	0	1	4 (3)	0	*A. hyperythra*
Sca	0	1	6 (0)	0	*A. hyperythra*
Ep	0	1	8 (6)	1	*A. hyperythra*
Loma	0	1	1 (1)	0	*A. hyperythra*
K23sjc	0	1	5 (3)	1	*A. hyperythra*
K46sjc	0	1	3 (1)	1	*A. hyperythra*
Teco	0	1	3 (1)	0	*A. hyperythra*
K90	0	1	3 (2)	0	*A. hyperythra*
K55	0	1	3 (2)	0	*A. hyperythra*
Con	0	1	4 (2)	0	*A. hyperythra*
Anc	0	1	5 (2)	0	*A. hyperythra*
Psm	0	1	5 (2)	0	*A. hyperythra*
Bal	0	1	5 (2)	0	*A. hyperythra*
Bal2	0	1	3 (0)	0	*A. hyperythra*
Car	0	1	2 (0)	0	*A. hyperythra*
Bar	0	1	3 (1)	0	*A. hyperythra*
Sas	0	1	2 (2)	7	*A. hyperythra*
Et	0	1	4 (4)	1	*A. hyperythra*
Plc	0	1	5 (3)	0	*A. hyperythra*
Ino	0	1	4 (2)	0	*A. hyperythra*
Ste	0	1	3 (1)	5	*A. hyperythra*
Rib	0	1	4 (3)	0	*A. hyperythra*
San	0	1	3 (1)	0	*A. hyperythra*
Bur	0	1	3 (0)	0	*A. hyperythra*
Cpul	0	1	3 (1)	0	*A. hyperythra*
Cnar	0	1	8 (1)	1	*A. hyperythra*
Gas	0	1	3 (1)	1	*A. hyperythra*
For	0	1	3 (1)	1	*A. hyperythra*
Mig	0	1	5 (3)	0	*A. hyperythra*
Csj	0	1	4 (1)	1	*A. hyperythra*
Csl	0	1	4 (2)	1	*A. hyperythra*

In the course of a phylogeographic study we captured live whiptails at 8 locations on 7 individual islands, as well as 35 peninsular locations (Fig. 1). As mentioned above, different components of antipredator behavior, such as vigilance, escape speed and hiding, are often considered separately. However, we have chosen to estimate the antipredator efficiency of the lizards directly, by acting ourselves as predators. To accomplish this, we chased each detected lizard until it was captured or lost (i.e., it disappeared into the groundcover or some other refuge). We then calculated the capturability (i.e., the inverse of ability to avoid predation) of whiptails at each sampling locality (See Methods Section).

**Figure 1:** The study area and the capture probability of lizards are showed. A. Study area. The Southern half of the Baja California peninsula and seven islands from Gulf of California. We visited 35 peninsular localities and eight on the islands.B. Capture probability of *A. hypertythra* lizards from 2004–2006 in Baja California. Data are least squares means (and 95% CL) from GLMM models controlling for locality and cat presence, back transformed to a probability using the inverse logit. The left panel refers to the analysis based on populations while the one on the right refers to the analysis focusing on the category of the species (insular endemic or not) present at each capture site.

## Results and Discussion

Most of the lizards chased on the 7 islands (58.2% , n = 146) were able to escape from the authors, while only 14.4% (n = 160) of those pursued on the peninsular mainland avoided capture. This indicates that, independent of local density, capturability was lower on the islands (*F*_(1, 261)_ = 13.86, *p* = 0.002; Fig. 1). Only at one of the 8 insular locations (San Francisco island) and 2 of the 35 peninsular locations (Sas and Ste), did the proportions of capture differ from the general pattern observed for insular or peninsular localities (Table 1).

The difficulty for the authors (i.e., predators) to capture lizards on the islands derived from the high wariness and efficient antipredator behavior of these animals. Although we did not measure these variables directly, insular lizards generally fled earlier and faster, and more often used underground refuges, than did peninsular mainland lizards. This higher wariness of insular lizards, which is presumably costly in terms of time, energy and opportunity, is surprising, given that insular animals are typically bolder and easier to capture due to the lack of many predators [14].

The wariness of insular lizards can increase following the introduction of foreign predators, such as domestic cats [7]. In our study area, cats are present on some islands, but were eradicated from others and were never present on San Francisco Island (Table 1). Lizards located on islands without cats managed to avoid capture in 66.0% of the chases (n = 50), while 54.1% (n = 96) escaped on islands with cats (Table 1). Thus, lizard wariness did not seem to increase at locations in which domestic cats are present. Expectedly, the presence of cats does not explain the differences we found in lizard capturability (*F*_(1,261)_ = 0.59; *p* = 0.44).

According to the “multi-predator hypothesis” [15], the presence of a single predator may be sufficient to explain the persistence of antipredator behavior in a given species. Thus, we should not expect tameness in insular whiptails, given that, due to their small body size, these animals can be prey for a number of island reptiles, birds and even some mammals. In fact, increased predation with respect to peninsular mainland populations could be occurring, thus explaining our results, if the number of alternative potential prey was reduced on the islands. Although criticized on occasion, the frequency of regenerated tails in lizard populations has long been considered an indirect estimator of predation pressure [16]. Therefore, we used the proportion of individual lizards with regenerated tails upon capture to test the hypothesis of higher predation intensity on the islands. Again, the results did not support this explanation, as the proportions are very similar between island locations (47.5% of the 61 captured lizards had regenerated tails) and those on the peninsular mainland (44.5% of the 137 captured lizards). Indeed, the proportion of lizards with regenerated tails within each locality did not influence their capturability (*F*_(1, 150)_ = 0.39, *p* = 0.53).

Conversely, the observed results may be related to a relative decrease of lizard wariness on the Baja California peninsula mainland. Although the islands are unpopulated, people inhabit the peninsular mainland, and thus whiptails in the latter area could be adaptively habituated to non-threatening stimuli coming from humans, given that the local population does not often pursue them. Supporting this contention is the fact that the lizards were relatively easy to capture on San José Island (Table 1), which was inhabited until recently. Habituation occurs when the magnitude of the antipredator response declines due to repeated non-threatening exposures to risk [17] (in this case to humans). However, we captured most of the peninsular animals at remote sites, very far of any human settlement (certainly, in many instances we were likely the first people that these short-lived lizards had encountered). Therefore, habituation to never-seen humans is unlikely to explain the difference in capturability observed for Orange-throated whiptails.

Likewise, it is possible that human populations acting as top predators could have generated a “mesopredator exclusion zone” [18] in the inhabited peninsula where small lizards would live under enemy-free conditions, thus becoming less wary. However, predation pressure, indirectly estimated from the proportion of regenerated tails, is similar for peninsular and insular lizard populations. Moreover, cats and dogs, which occasionally prey on lizards, are often found living near human settlements. Finally, the Baja California peninsula is sparsely populated, as previously noted, and a relative high human density would be necessary to produce the mentioned predator exclusion zone.

The results of our study suggest that antipredator behavior of insular lizards is more efficient than that of mainland ones, and that the frequently cited reason, namely higher “natural” predation pressure, does not explain this observation. Nevertheless we can contemplate another cause. As lizards generally respond to predator-specific cues [19], the wariness of *Aspidoscelis* spp. on islands might be related to the perception of human-derived risk. This proposition may appear counterintuitive, given that we have previously mentioned that the islands are uninhabited. However, insular species are attractive for collectors. For example, insular *Aspidoscelis* specimens preserved in officially sanctioned collections seem to be quite numerous. In only two published papers, 160 specimens from Carmen Island, 110 from San José, 85 from Espíritu Santo-Partida, 80 from Cerralvo, 68 from Montserrat, 65 from San Francisco and 47 from Coronados were studied [20], [12]. Although lizards from the Baja California peninsula mainland are also abundant in scientific collections, the number of collected specimens per unit surface area is negligible. Furthermore, it can be presumed that scientific collectors will be particularly attracted to insular endemics, which should be warier. In fact, individuals of island-specific endemic species are less capturable than those belonging to the nominal species (*F*_(1,261)_ = 14.8; *p* = 0.0002; Fig. 1).

In addition to officially sanctioned specimen collection, occasional illegal harvesting may also be important. Illegal collection and trafficking of reptiles from the Gulf of California is a well-known phenomenon and a particular risk has been suggested for insular endemic species [21, and references therein]. For some species a commercial demand can be expected from pet owners, but insular lizards of the *Aspidoscelis* group lack commercial value and it is nearly impossible for non-specialists to differentiate between them at species-level. Consequently, we believe that the demand may come specifically from academic-related collectors, given that species from the Gulf of California make good case studies of speciation and island biogeography. In fact, local fishermen have informed us of the relatively frequent groups of students who rent boats to travel to the various islands for the study (and presumably collection) of spiders, beetles, lizards and other animals.

Is the observed wariness of insular lizards learnt or innate behavior? Long-lived reptiles learn to recognize risk and increase their wariness after stressful experiences [22], but for short-lived Orange-throated whiptails differences in the ability to avoid capture must be genetically based, implying a rapid evolution of antipredator behavior. Most islands in the Gulf of California are quite small and whiptails live only on flat areas with sandy soils, a habitat restricted to the proximity of inlets (where collectors, such as the authors, predominately arrive). Thus, low population numbers, combined with a limited number of suitable places for specimen collection, favours an intense predation pressure selecting for warier individuals. Additionally, whiptails have a short generation time and visits by prospective collectors are infrequent, and consequently, for an individual lizard the opportunities to learn escape behaviors are reduced. Natural selection explains genetically-based differences in the wariness of another whiptail species, *Aspidoscelis tesselata* [10], and similar laboratory experiments could be used with Orange-throated whiptails to support our contention. Moreover, harvest-induced phenotypic changes seem to accumulate unusually quickly [23].

Our suggestion that there is a relationship between lizard antipredator behavior and human harvesting is a hypothesis that we cannot test with the available data as visits to the islands were not quantified and a single significant collection visit, even some years ago, could have produced selection effects on a small population. However, this lack of complete certainty is frequent in conservation biology, which, since its origins, identified the risks of the so-called “Nero dilemma”: choosing to do nothing rather than advancing a possibly flawed hypothesis [24]. Indeed, teaching evolution and investigating taxonomic and systematic issues play an important role in the global fight for the conservation of biodiversity, but it is also obvious that tensions with conservationists can arise [e.g., 25]. Several examples from Mexico, as noted by Rodríguez-Estrella and Blázquez [26], confirm the risks of excessive specimen collection. First, three freshwater fish species of the genus *Cyprinodon*, restricted to a few ponds in Nuevo León, were described in 1984 and then quickly exterminated in 1986, 1990 and 1994 after important collection activities. Second, the elf-owl (*Micrathene witheyi socorroensis*) from Socorro Island, in the Revillagigedo Archipelago, which was collected every time naturalists visited the island, was last recorded (and collected) in 1932. Third, the last record sighting in the wild of the endemic dove species from Socorro Island (*Zenaidura graysone*) occurred in 1958; although now it is known that some of the last individuals were live-collected in secrecy and are at present bred in captivity. Even more interesting is the fact that specimen collection was traditionally a competitive activity, so that in some cases particular morphs were purposefully over-collected because they were more valuable when they became rarer [27].

A dual-use dilemma arises when the same piece of scientific research has the potential to be used for harm as well as for good [28]. Dual-use dilemmas have been identified for taxonomists describing commercially valuable new species [3]. The results of the present study underscore the ability of behavioral studies to identify a possible dilemma resulting from the increased value of restricted taxonomic entities as scientific commodities.

## Materials and Methods

All lizards were chased and captured in the same way by the same group of people (four of the authors -MD, MCB, LS and JAG- and A Cota). Typically, lizards of the *Aspidoscelis hyperythra* group are active wanderers, moving in the open while looking for prey. In order to capture specimens, we walked slowly over the designated search area scanning the ground carefully until a lizard was detected. We made an effort not to disturb the target individual once it had been identified, however, most of the time it ran under a nearby bush. All of us then surrounded the bush and attempted to locate the animal underneath and subsequently snare it with a noose (a thread loop at the end of a rod) around the neck. The lizards could disappear (e.g., into a hole in the ground) or were captured almost immediately. However, it was also possible for an individual to move to one or more different bushes before it was ensnared or lost. Thus, for each individual the process lasted from several seconds to a few minutes.

Field research took place during the month of September in 2004 and 2005 and May 2006. The search and capture of lizards was carried out from approximately 9:00 to 17:00 hours, but the time devoted to every individual and each locality depended on the ability of the animals to escape and their abundance and activity level (inactive lizards were not detected). Typically, each day we captured lizards at two or three locations on the peninsular mainland and one insular location. We visited each locality only once over the course of the study. Each of the authors made his own thread noose whenever it was needed (usually several times a day). Lizard noosing was made by the collector closest to the animal, and all of us had prior experience catching lizards using this method.

In the field, for each captured lizard we noted morphological characteristics and collected a 1****cm segment from the end of its tail for DNA analyses. This short section represents a very small portion of the extremely long and thin tail of this species. Furthermore, as with many lizard species, whiptails have the ability for tail-autotomy and posterior regeneration, and thus the loss of 1****cm of their tail tip is not harmful to the animals. We carefully clipped the tail tip with a scalpel disinfected with ethanol and we then applied a piece of cotton with ethanol to the cut. All lizards were released in the shadow of a bush a short time after capture. Permissions for this sampling protocol were obtained from the environmental authority in Mexico (SEMARNAT permit number # 11311); the protocol also conforms to the policies of the ethics committees of our institutions.

Data were analysed with GLMM models [29]. Capturability was used as the response variable and endemicity, presence of domestic cats and percentage of captured lizards with regenerated tails as explanatory variables. Locality was used as a random factor. For the present study, we define capturability as the relationship between the number of effective individuals captured and the number of lizards we tried to ensnare at each sampling locality. In this way, the bias of differential abundance or activity level between areas was avoided. We did not consider the initial habitat where each lizard was discovered given that virtually all individuals ran under a bush immediately upon detection.
